# Asiatic acid re-sensitizes multidrug-resistant A549/DDP cells to cisplatin by down regulating long non-coding RNA metastasis associated lung adenocarcinoma transcript 1/β-catenin signaling

This article has been retracted.

**DOI:** 10.1080/21655979.2022.2079302

**Published:** 2022-05-24

**Authors:** Qilai Cheng, Shanshan Zhang, Bing Zhong, Zhixi Chen, Fang Peng

**Affiliations:** a College of Pharmacy, Gannan Medical University, Ganzhou, Jiangxi, China; b Department of Pharmacy, First Affiliated Hospital of Gannan Medical University, Ganzhou, Jiangxi, China; c Department of Pathology, Ganzhou People’s Hospital, Ganzhou, Jiangxi, China

**Keywords:** Asiatic acid, drug resistance, A549/DDP cells, MALAT1, miR-1297, β-catenin

## Abstract

Drug resistance becomes a challenge in the therapeutic management of non-small cell lung cancer (NSCLC). According to our former research, asiatic acid (AA) re-sensitized A549/DDP cells to cisplatin (DDP) through decreasing multidrug resistance protein 1 (MDR1) expression level. However, the relevant underlying mechanisms are still unclear. Long non-coding RNA (lncRNA) MALAT1 shows close association with chemo-resistance. As reported in this research, AA increased apoptosis rate, down regulated the expression of MALAT1, p300, β-catenin, and MDR1, up regulated the expression of miR-1297, and decreased β-catenin nuclear translocation in A549/DDP cells. MALAT1 knockdown expression abolished the drug resistance of A549/DDP cells and increased cell apoptosis. MALAT1 could potentially produce interactions with miR-1297, which targeted to degradation of p300. In addition, p300 overexpression effectively rescued the effects of MALAT1 knockdown expression on A549/DDP cells and activate the expression of β-catenin/MDR1 signaling, and these could be effectively blocked by AA treatment. Conclusively, AA could re-sensitize A549/DDP cells to DDP through down-regulating MALAT1/miR-1297/p300/β-catenin signaling.

## Highlights

- MALAT1 promoted the drug resistance of A549/DDP cells.
- MALAT1 activated p300/β-catenin by sponging miR-1297.
- AA re-sensitized A549/DDP cells by inhibiting MALAT1/p300/β-catenin signaling.

## 1. Introduction

Non-small cell lung cancer (NSCLC), a highly frequent lung cancer (LC) in humans featuring high mortality, makes up around 85% of overall lung cancer cases [1]. In clinic, most patients with NSCLC at the advanced stage are diagnosed for their first visit, rendering poor prognosis [2]. Chemotherapy, as the mainstream therapy for management of advanced NSCLC, often causes chemoresistance and series of adverse effects. For example, cisplatin (DDP) is often applied as a first-line drug to manage NSCLC. Although DDP demonstrates good efficacy in treating NSCLC, its clinical application is usually constrained by the occurrence of drug resistance [3]. It is an urgent issue that needs to be addressed. However, potential DDP resistance mechanisms remain sophisticated.

Canonical Wnt/β-catenin signaling is correlated with normal embryonic development as well as cancerous cell survival. The activity is mediated by the expression, localization, acetylation, and phosphorylation of β-catenin [4]. Research reports the significant increase of β-catenin expression in DDP-resistant NSCLC cells [5]. DDP activates Wnt/β-catenin signaling by a ligand-independent regulatory mechanism, and inhibition of β-catenin expression can effectively reverse DDP resistance in DDP-treated mice models [6]. Multidrug resistance protein 1 (MDR1) is a transmembrane protein, which can transport chemotherapeutic agents in various structures outward energy-dependently. The overexpression of MDR1 after chemotherapy results in drug resistance [7]. β-catenin signaling activation targets to increase MDR1 expression by binding to its promoter [8]. Thus, Wnt/β-catenin signaling becomes an underlying target of therapeutic management of drug resistance.

Long non-coding RNAs (lncRNAs) represent the RNA transcripts that are more than 200 nucleotides in length encoded by endogenous genes. LncRNAs have been implicated in the regulation of gene level through post-transcriptional, transcriptional modulation, and epigenetic modification. Metastasis-related lung adenocarcinoma transcript 1 (MALAT1) has been firstly recognized in NSCLC [9]. Its primary sequence includes over 8000 bp, which is highly conserved across 33 mammalian species [10]. MALAT1 expression can be found from nearly overall human tissues, reaching its peak in pancreas and lung [11]. MALAT1 is found to facilitate human cancer and chemoresistance development [12]. For DDP-resistant A549/DDP cells, increased MALAT1 expression promotes the activity of MDR1 through activation of signal transducer and activator of transcription 3 (STAT3) signaling, leading to decreased sensitivity to DDP and a potently poor prognosis [3]. Many reports have proved the role of MALAT1 in up-regulating the activity of β-catenin signaling [13,14]. However, whether MALAT1 contributes to the drug resistance of A549/DDP cells to DDP through mediating β-catenin/MDR1 axis is still unclear.

Asiatic acid (AA) is a triterpenoid isolated in *Centella asiatica*, a traditional Chinese medicine. AA possesses the protective activity in anti-cancers, anti-inflammation, anti-oxidation, and hepatoprotection [15,16]. It has been reported that AA can suppress the growth of tongue cancer by induction of endoplasmic reticulum (ER) stress and activation of Calpain and GRP78/IRE1α/JNK pathways [17]. AA inhibits the invasion and proliferation of breast [18], lung [19], and bile duct [20] cancers. The inhibitory effects of AA against various cancers have been reviewed [21]. AA also ameliorates drug resistance in cancers. It is well documented that AA is the activator for Smad7, which serves as the negative regulator for NF-κB pathway [22]. NF-κB pathway activation can mediate p-glycoprotein expression, a key factor of multidrug resistance [23]. In DDP-resistant nasopharyngeal carcinoma cells, AA promotes cell apoptosis by activating p38 MAPK signaling [24]. To explore the possible underlying mechanism of AA in re-sensitizing A549/DDP cells to DDP, we mainly study whether AA re-sensitizes A549/DDP cells to DDP by down regulating LncRNA MALAT1/β-catenin signaling.

## 2. Materials and methods

### 2.1. General

Experimental profiles gain approval (NO.2020015) from Ethics Committee in Gannan Medical University based on Declaration of Helsinki Principles. AA (≥98%; Cat.no.A2612), DDP (Cat.no.1134357), DMSO (Cat.no.D8418), anti-immunoglobulin G (anti-IgG; Cat.no.I5131) and anti-argonaute2 antibody (anti-Ago2; Cat.no.MABE56) were provided by Sigma-Aldrich (St. Louis, MO, USA). The antibodies of TCF4 (Cat.no.2569), β-catenin (Cat.no.8480), MDR1 (Cat.no.13342), p300 (Cat.no.86377), cleaved caspase-3 (Cat.no.9661), caspase-3 (Cat.no.9662), and GAPDH (Cat.no.5174) were provided by Cell Signaling Technology (Danvers, MA, USA). TUNEL kits (Cat.no.C1088) and horseradish peroxidase-conjugated IgG (Cat.no.A0201) were acquired from Beyotime (Shanghai, China).

### 2.2. Cell culture

Human lung adenocarcinoma (LUAD) A549 cells together with DDP-resistant A549/DDP cells were obtained from ATCC (Manassas, VA, USA). RPMI-1640 medium (Gibco, Waltham, MA, USA) with 1% penicillin/streptomycin (Invitrogen) and 10% fetal bovine serum (FBS) (Invitrogen, Carlsbad, CA, USA) was used in cell cultivation. Cells were cultured under 5% CO2 and 37°C conditions. Cells were utilized at exponential stage for experiment.

### 2.3. Cell transfection

The synthesis of three short-hairpin RNAs (shRNAs) (sh-MALAT1-1/-2/-3) together with the scrambled shRNA control (sh-NC) was performed at Hibio Tech Co., Ltd (Hangzhou, China). The shRNAs were introduced to pGPH1/Neo (Hibio, Hangzhou, China), followed by transfection in A549 or A549/DDP cells via lipofectamine 2000 (Invitrogen). Neomycin (Sigma-Aldrich, Cat.no.1405–10-3) was used to screen the stable transfectants [25].

miR-1297 mimics together with the corresponding NC (miR-NC) was provided by RiboBio (Guangzhou, China). A549 or A549/DDP cells that achieved 60% confluency (1 × 10^5^ cells/well) was applied to transfection by lipofectamine 2000 (Invitrogen), and then cultivated in a day using 6-well plates. The concentrations of miR-1297 mimics as well as miR-NC in the eventual transfection system were set at 50 nM [26].

In addition, we constructed pcDNA3.1-p300 vector (RiboBio) through the clone of p300ʹs open reading frame (ORF) in pcDNA3.1 vector. Afterward, we used lipofectamine 2000 (Invitrogen) to transfect pcDNA3.1-p300 vectors in A549 or A549/DDP cells [26].

### 2.4. MTT assays

After transfection, we cultivated A549 or A549/DDP cells (5 × 10^3^/well) at 37°C for 48 h. Assays were performed following the kit specifications (Cat.no.C0009S) (Beyotime). MTT (0.5 mg/mL) was added for co-incubating cells under 37°C for 4 h. Afterward, 150 μL DMSO was introduced for dissolving the formazan in the darkness. The wavelength of 490 nm was calculated using the microplate reader (Thermo Fisher Scientific).

### 2.5. Apoptosis assay

Flow cytometry (FCM, FACSCalibur BD, San Jose, CA, USA) was adopted to determine apoptotic changes with Annexin V-FITC apoptosis assay, following kit specifications (Cat.no.C1062L) (Beyotime). Briefly, cells were harvested and cultured with buffer and Annexin V-FITC as well as PI. Alterations of cell apoptosis were observed.

### 2.6. qRT-PCR

Trizol reagent (Invitrogen) was used to extract total RNA following kit specifications. Meanwhile, 2 μg RNA was collected to prepare cDNA through reverse transcription via M-MLV (Promega, Madison, WI, USA). Thereafter, qRT-PCR assays via Power SYBRs Green PCR Master Mix (Applied Biosystems, CA, USA) were performed for detecting the expression levels of MALAT1, β-catenin, caspase-3, TCF4, and p300. The miR-1297 expression with Taqman Universal Master Mix II kit and Taqman MicroRNA Reverse Transcription Kit (Applied Biosystems) was tested. U6 and GAPDH served as endogenous references of miRNA and mRNA. The sense/anti-sense chain primers based on Biomics were acquired. Table 1 shows the primer sequences. miR-1297 and mRNAs gene expression was denoted as fold changes using 2^−ΔΔCT^ method [27].

**Table 1.** Primer sequences for different genes

Genes	Primers	Sequences (5’-3’)
MALAT1	Forward	TGGGGGAGTTTCGTACTGAG
	Reverse	TCTCCAGGACTTGGCAGTCT
β-catenin	Forward	AAAGCGGCTGTTAGTCACTGG
	Reverse	CGAGTCATTGCATACTGTCCAT
TCF4	Forward	CCTGGCTATGCAGGAATGTT
	Reverse	CAGGAGGCGTACAGGAAGAG
p300	Forward	CTTCCCCACTGTCGCACAAT
	Reverse	TTTGTCGAGAAGATGCACAGTGT
Caspase-3	Forward	TTTGTTTGTGTGCTTCTGAGCC
	Reverse	ATTCTGTTGCCACCTTTCGG
GAPDH	Forward	CATGTTCCAATATGATTCCACC
	Reverse	GATGGGATTTCCATTGATGAC
miR-1297	Forward	TCGGCAGGTTCAAGTAATT
	Reverse	CTCAACTGGTGTCGTGGA
U6	Forward	ATTGGAACGATACAGAGAAGATT
	Reverse	GGAACGCTTCACGAATTTG

### 2.7. Western-blot (WB) assay

Total proteins were retrieved with pre-chilled RIPA lysis buffer (Beyotime), and the protein concentration was analyzed with BCA protein assay, following specific instructions (Cat.no.P0010) (Beyotime). Total proteins (30 μg) in every group underwent 10% SDS-PAGE, followed by transfer to PVDF membranes (Millipore, Burlington, MA, USA). Upon blocking within TBS that containing 5% skimmed milk powder under ambient temperature for 1 h, β-catenin (1:1,000; Cell Signaling Technology), TCF4 (1:1,000; Cell Signaling Technology), p300 (1:1,000; Cell Signaling Technology), caspase-3 (1:1,000; Cell Signaling Technology), cleaved caspase-3 (1:1,000; Cell Signaling Technology), as well as GAPDH (1:1,000; Cell Signaling Technology) primary antibodies were cultured overnight under 4°C. Afterward, membranes were cultured using HRP-labeled secondary antibody (1:2,000) for 1 h. The protein bands were tested with Quantity One software v4.6.2 (Bio-Rad) and ECL assay system (Bio-Rad, Hercules, CA, USA).

### 2.8. Dual-luciferase reporter assay

TargetScan7.2 (http://www.targetscan.org) and StarBase v2.0 (http://starbase.sysu.edu.cn) were adopted for seeking target genes of miR-1297 and miRNA targets of MALAT1, separately. Recombinant luciferase plasmids were established through the clone of 3’-UTR of p300 and wild-type (WT) MALAT1 in pGL-3 luciferase basic vector (Promega). Additionally, the mutant (MUT) types containing miR-1297ʹs mutant binding sites as MUT-p300 and MUT-MALAT1 were constructed. Later, every established plasmid was transfected in A549 or A549/DDP cells using miR-NC or miR-1297 mimics via lipofectamine 2000 (Invitrogen). After 48-hour culture under 37°C, firefly/Renilla luciferase activities were analyzed with Glomax 96 luminometer (Promega), following specific instructions. Firefly luciferase reporter was normalized to the luciferase activity of Renilla [25].

### 2.9. RNA immunoprecipitation (RIP) assays

RIP assays were conducted for exploring the direct interplay between MALAT1 and miR-1297 with Magna RIP kit (EMD Millipore), following kit specifications. Centrifugation of A549 or A549/DDP cells was conducted under 15000 × g and 4°C for a 10-min period. Later, A549 or A549/DDP cells (2 × 10^7^ cells) were lysed in RIPA lysis buffer (Beyotime). Subsequently, cells were cultured using magnetic beads pre-coated by anti-Ago2 and anti-IgG antibodies (1:150) for NC. RNA was extracted with TRIzol reagent (Invitrogen), then the RNA level was tested using qRT-PCR. Eventually, the expression levels of MALAT1 and miR-1297 levels, respectively, in anti-Ago2 and anti-IgG groups were compared [25].

### 2.10. Immunofluorescence (IF) assay

A549 or A549/DDP cells were fastened using 4% paraformaldehyde. 0.1% Triton X-100 was adopted for infiltrating nuclear membrane and cells. Next, cells were blocked with 5% protease-free bovine serum albumin (BSA), washed in PBS, and cultured using primary antibody overnight under 4°C. Cells were rinsed in PBS, then cultured using fluorescein-conjugated goat anti-human IgG antibody under ambient temperature for 1 h. Then, cells were placed within the medium with DAPI upon being rinsed in PBS. Afterward, the slides were observed with confocal laser scanning microscope (Leica Microsystems), and the corresponding fluorescence intensity was tested with ImageJ software 2.1 (Bethesda, MD, USA) [28].

### 2.11. Statistical analysis

Each experiment was conducted in triplicate, and results were denoted in a form of mean ± SEM. SPSS20.0 (IBM Corp., Armonk, New York, USA) was applied in statistical analyses. Differences across groups were compared by one-way ANOVA as well as Tukey’s post hoc test. Meanwhile, the unpaired Student’s t-test was adopted to compare statistics in both groups. P < 0.05 stood for statistical significance.

## 3. Results

The roles of MALAT1 in many cancers and chemoresistance have been investigated. However, its role in the drug resistance of A549/DDP cells is still unknown. AA has been reported the anti-cancer activity. Whether AA exhibits protective against the drug resistance of A549/DDP cells still needs to be elucidated. In this study, we found that knockdown of MALAT1 expression ameliorated the drug resistance of A549/DDP cells by sponging miR-1297, which targets to degrade p300. AA could significantly re-sensitize A549/DDP cells by inhibiting the expression of MALAT1/miR-1297/p300 signaling, blocking the activity of β-catenin pathway.

### 3.1. AA increased apoptosis and decreased MALAT1/β-catenin pathway activation within A549/DDP cells

As results in Figure 1 (a) and (b), combined treatment with DDP (1.0 μg/mL) and AA significantly triggered apoptosis of A549 cells and A549/DDP cells. A549 cells rather than A549/DDP cells showed DDP sensitivity, as indicated through decreased expression of MALAT1 (Figure 1(c)), β-catenin (Figure 1 (d, i, j, and k)), p300 (Figure 1(e, i and l)), and MDR1 (figure 1 (f, i and m)) and increased expression of caspase-3 (Figure 1 (g, i and n)) and miR-1297 (Figure 1(h)). The protein expression of β-catenin in the cytoplasm by treatment with DDP+AA was significantly increased than that in the nucleus (Figure 1 (j) and (k)). Similarly, the nuclear expression for β-catenin was remarkably decreased by treatment with DDP+AA. The cleaved caspase-3 expression (Figure 1 (i) and (o)) was greatly enhanced by combined treatment with DDP and AA. Immunofluorescence assay (Figure 1(p)) showed that β-catenin located in A549/DDP cell nucleus, in contrast to that in A549 cell cytoplasm. These indicated that A549/DDP showed DDP resistance. DDP plus AA treatment re-sensitized A549/DDP cells to DDP, as indicated by increased apoptosis ratio, enhanced MALAT1/β-catenin signaling expression, and β-catenin re-location to the cytoplasm.

**Figure 1.** AA increased apoptosis and decreased the expression of MALAT1/β-catenin signaling in A549/DDP cells. (a) Cell apoptosis was tested using flow cytometer. (b) The apoptosis rate was calculated. MALAT1 (c), β-catenin (d), p300 (e), MDR1 (f), caspase-3 (g), and miR-1297 (h) gene levels were tested by qRT-PCR. Protein levels were tested by WB assay (i). Fold changes in cytoplasmic (j) and nuclear (k) β-catenin, p300 (l), MDR1 (m), caspase-3 (n), and cleaved caspase-3 (o) expression were calculated. (p) The subcellular location of β-catenin was analyzed through immunofluorescence assays (×400 magnification). The experiments were conducted three times independently, with data denoted as mean ± SD. *P < 0.05, **P < 0.01.

### 3.2. Knockdown expression of MALAT1 ameliorated A549/DDP cells’ drug resistance

For investigating the effects of MALAT1 on DDP-treated A549/DDP cells, three shRNAs against MALAT1 were synthesized and employed to knockdown MALAT1 expression by transfection. qRT-PCR analysis was conducted for confirming the efficiency (Figure 2(a)). The shRNAs showed significantly inhibitory activity against MALAT1 expression of A549/DDP cells, and sh-MALAT1-2 exhibited the most efficiency. Thus, sh-MALAT1-2 was selected for the following experiments. Sh-MALAT1 transfection remarkably lowered the viability of A549/DDP cells, compared with sh-NC (Figure 2(b)). Knockdown expression of MALAT1 increased the apoptosis rate (Figure 2(c,d)) and inhibited β-catenin nuclear translocation (Figure 2(e)) of DDP-treated A549/DDP cells. Collectively, MALAT1 expression was correlated with the drug resistance of A549/DDP cells.

**Figure 2.** MALAT1 silencing mitigated the drug resistance of A549/DDP cells. (a) sh-MALAT1 silencing efficiency was measured using qRT-PCR. (b) MTT assays were conducted for detecting cell viability. (c) Flow cytometer was performed to test cell apoptosis. (d) The apoptosis rate was measured. (e) The subcellular location of β-catenin was detected through immunofluorescence assays (×400 magnification). The experiments were conducted three times independently, with data denoted as mean ±SD. *P < 0.05, **P < 0.01.

### 3.3. MALAT1 interacted with miR-1297

For investigating the biological functions of MALAT1 in DDP-treated A549/DDP cells, the potential miRNA that bound to MALAT1 was predicted using Starbase2.0 software. Results showed that miR-1297 was predicted to be the underlying target for MALAT1 (Figure 3(a)). According to dual-luciferase reporter assays, WT-MALAT1 reporter luciferase activity reduced by over 60% (Figure 3(b)). Comparatively, the luciferase activity of MUT-MALAT1 reporter and NC reporter groups did not show any significant difference. RIP assays showed the interplay between MALAT1 and miR-1297 in A549/DDP cells (Figure 3(c)). Collectively, miR-1297 was an underlying target for MALAT1.

**Figure 3.** MiR-1297 was a potential target for MALAT1. (a) The underlying interaction of MALAT1 with miR-1297 was tested using Starbase2.0. (b) Relative luciferase activities were tested for A549/DDP cells after WT/MUT-MALAT1 co-transfection with miR-1297 mimics/miR-NC. Association of MALAT1 with miR-1297 was determined through RIP assay. The experiments were conducted three times independently, with data denoted as mean ± SD. *P < 0.05, **P < 0.01.

### 3.4. Overexpression of miR-1297 inhibited the effects of MALAT1 on A549/DDP cells

For exploring miR-1297ʹs effects on A549/DDP cells, miR-1297 mimics were transfected in A549/DDP cells. Then, qRT-PCR was conducted for detecting miR-1297 expression for verification of successful transfection (Figure 4(a)). miR-1297 overexpression inhibited MALAT1 expression (Figure 4(b)), increased apoptosis rate (Figure 4(c,d)), and inhibited β-catenin nuclear translocation (Figure 4(e)) in A549/DDP cells. Collectively, miR-1297 overexpression could abrogate the impacts of MALAT1 on A549/DDP cells.

**Figure 4.** miR-1297 over-expression inhibited the impact of MALAT1 impact on A549/DDP cells. miR-1297 (a) and MALAT1 (b) levels were measured through qRT-PCR within A549/DDP cells after transfection with miR-1297 mimics. (c) Cell apoptosis was tested using Flow cytometer. (d) Apoptosis rate was measured. (e) The subcellular location of β-catenin was detected through immunofluorescence assays (×400 magnification). The experiments were conducted three times independently, with data denoted as mean ±SD. *P < 0.05 and **P < 0.01.

### 3.5. P300 served as miR-1297ʹs target

For investigating how miR-1297 influenced A549/DDP cells in biological actions, TargetScan7.2 was adopted for predicting the underlying target for miR-1297. Results showed miR-1297 could bind to the 3’-UTR of p300 (Figure 5(a)). As indicated by dual-luciferase reporter assays, WT-p300 luciferase activity decreased by over 60%. In contrast, difference in luciferase activity was not significant between MUT-p300 and NC reporters. In miR-1297 mimics-transfected A549/DDP cells, the mRNA and protein expression of p300 were significantly down regulated. Thus, miR-1297 might specifically target to degrade p300.

**Figure 5.** P300 served as a target of miR-1297. (a) The underlying interaction of miR-1297 with p300 was tested using TargetScan7.2. (b) Relative luciferase activities were tested for A549/DDP cells after WT/MUT-p300 co-transfection with miR-1297 mimics/miR-NC. P300 mRNA (c) and the protein (d-e) levels were tested in A549/DDP cells after miR-1297/miR-NC transfection. Each experiment was conducted three times independently, with data denoted as mean ±SD. *P < 0.05, **P < 0.01.

### 3.6. AA enhanced DDP sensitivity of A549/DDP cells by regulating MALAT1/miR-1297/p300 signaling

To explore the molecular mechanisms for AA in re-sensitizing A549/DDP to DDP, sh-MALAT1 and pcDNA3.1-p300 were co-transfected into A549/DDP cells. The expression of MALAT1 (Figure 6(a)) and p300 (Figure 6(a–c)) were tested, proving that transfection succeeded. According to the findings, p300 overexpression could effectively reserve the effects induced by MALAT1 knockdown expression, as shown by increased expression of β-catenin (Figure 6 (d, g, and h)) and MDR1 (Figure 6(e, g, and i)), decreased expression of caspase-3 (figure 6(f, g, and j)) and cleaved caspase-3 expression (Figure 6 (g) and (k)), and decreased apoptotic ratio (Figure 6 (l) and (m)) and β-catenin nuclear location (Figure 6(n)) in A549/DDP cells. However, AA administration could ameliorate the biological activities of p300 overexpression. Collectively, AA re-sensitized A549/DDP cells to DDP through regulating MALAT1/miR-1297/p300 signaling.

**Figure 6.** AA re-sensitized A549/DDP cells to DDP through regulating MALAT1/miR-1297/p300 signaling. (a) The expression of MALAT1 and p300 in co-transfection of sh-MALAT1 and pcDNA3.1-p300 into A549/DDP cells was tested using qRT-PCR. (b-c) p300 protein expression was tested. β-catenin (d), MDR1 (e), and caspase-3 (f) gene expression was tested using qRT-PCR. β-catenin (g, h), MDR1 (g, i), caspase-3 (g, j), and cleaved caspase-3 (g, k) protein expression was tested using Western Blot. (l) Cell apoptosis was measured through Flow cytometer. (m) Analysis of apoptosis rate. (n) The subcellular location of β-catenin was detected through immunofluorescence assays (×400 magnification). The experiments were conducted three times independently, with data denoted as mean ±SD. *P < 0.05, **P < 0.01.

## 4. Discussion

Drug resistance presents the leading challenge to cancer clinical therapeutic management. Many pre-clinical reports have shown that DDP resistance of lung cancers results from some aberrant signaling activation, including Wnt signaling [5,29]. The drug resistance development mechanisms in lung cancers remain to be fully elucidated. LncRNAs are verified to contribute to regulating the drug resistance in different cancers [30]. According to this study, AA effectively ameliorated DDP drug resistance of A549/DDP cells. Additionally, AA decreased lncRNA MALAT1/miR-1297/p300 signaling activity. Knockdown expression of MALAT1 reversed the drug resistance of A549/DDP cells to DDP. MALAT1 potentially interacted with miR-1297, which targeted to degradation of p300. p300 overexpression led to activation of β-catenin/MDR1 signaling. Collectively, AA enhanced the sensitivity of A549/DDP cells to DDP through decreasing MALAT1/p300 expression through sponging miR-1297. Possibly, there existed a synergistic effect between AA and DDP. Further investigation is still needed to clarify.

MALAT1 is an oncogene with high conservation degree, which promotes cancer development and regulates radio-sensitivity and chemo-sensitivity in cancer cells [9,31]. MALAT1 has been considered as the prognostic cytokine that initially marked to be the survival marker, due to that it is related to tumor migration, metastasis, and recurrence among NSCLC patients [10]. Recently, multiple studies on the roles of MALAT1 in NSCLC have been reported. MALAT1 has been greatly overexpressed in NSCLC and is significantly associated proliferation, metastasis, and decreased apoptosis in NSCLC cells by regulating miR-185/MDM4 signaling [32]. Knockdown expression of MALAT1 ameliorates the growth, invasion, and metastasis and increases apoptosis through mediating miR-515/TRIM65 axis [33]. As shown in this study, MALAT1 expression significantly increased within A549/DDP cells. Knockdown expression of MALAT1 by transfection with sh-MALAT1 increased the apoptosis rate, ameliorating the drug resistance of A549/DDP cells.

β-catenin-triggered classical Wnt pathway has been accepted to be the crucial regulating factor for chemo-resistance, and suppressing Wnt/β-catenin pathway enhances sensitivity to chemo-therapeutic agents in prostate cancer [34]. Wnt/β-catenin pathway activation is associated with Oct4/Nanog-mediated epithelial-mesenchymal transition (EMT) and drug resistance, and silencing β-catenin abrogates Oct4/Nanog’s effects on NSCLC cells, effectively reversing the drug resistance [35]. In the activated Wnt/β-catenin pathway, un-phosphorylated β-catenin induces stability and translocation into the nucleus to form a complex with TCF4/LEF1, resulting in up regulation of target genes transcription [36]. MDR1 has been proved to be a downstream target for Wnt/β-catenin signaling [37]. MDR1 overexpression increases the drug efflux and is related to multidrug resistance [38]. According to this study, DDP-resistant A549/DDP cells exhibited high expression for β-catenin and MDR1, nuclear translocation of β-catenin, and decreased apoptosis rate. These indicated that the β-catenin/MDR1 signaling in A549/DDP cells was activated.

P300 is a transcriptional co-factor of β-catenin. P300/β-catenin complex plays a critical role in activating β-catenin in the transcriptional activity [39]. The distal N-termini of p300 recruit members from different nuclear receptor families through the LXXLL motif, facilitating the transcriptional activity of β-catenin [40]. It has been reported that p300 has histone acetyltransferase (HAT) activity, promoting APE1/YB-1/p300 complex to bind to MDR1 promoter [41]. Acetylation and deacetylation regulate the stability of β-catenin. Formation a complex of p300 with β-catenin may increase its stability and nuclear distribution and enhance β-catenin/LEF1-mediated transcriptional activity [42].

In addition, p300 was considered a direct target for miR-1297, which was sponged by MALAT1. Knockdown expression of MALAT1-induced up-regulation of miR-1297 expression, down-regulation of p300 expression, as well as decreased nuclear translocation of β-catenin. Similarly, miR-1297 mimics transfection also down regulated the expression of p300 and decreased nuclear translocation of β-catenin. Reversely, p300 overexpression rescued the effects of MALAT1 knockdown expression on A549/DDP cells after sh-MALAT1 co-transfection with pcDNA3.1-p300, as shown by increased nuclear translocation for β-catenin, up regulated expression for MDR1, as well as decreased apoptosis rate. All the data suggested that MALAT1 increased the drug resistance by mediating β-catenin/MDR1 signaling through miR-1297/p300 axis in A549/DDP cells.

AA has been recently proved to exhibit anti-fungal effects and inhibit drug efflux pump activity, showing great potential in overcoming the drug resistance of *Candida albicans* [43]. The anti-cancer effects of AA have been comprehensively reviewed [21]. AA has been showed the cytotoxicity and negatively regulated Bcl-2 expression of A549 cells through up-regulation of miR-1290 expression [44]. NF-κB activates Wnt/β-catenin pathway expression within tumors [45,46]. The crosstalk between MAPK and Wnt/β-catenin pathway has been reported [47,48]. From this study, we found that AA effectively down-regulated MALAT1 and β-catenin/MDR1 signaling expression and increased apoptosis of A549/DDP cells.

There are still some limitations in this study. Nuclear and cytoplasmic β-catenin levels were studied using WB and immunofluorescence assays. Disappointedly, β-catenin expression within A549/DDP cells determined by immunofluorescence assays was not consistent with that detected by western blot assays. The factors influencing it might be various, including the experimental condition, the investigators, or the machine. A549/DDP cell was the only one single-cell line to be studied, and this might produce controversial. It is essential to investigate how AA interacts with cells and how AA comes across the cellular membrane. Natural products have been reported to reverse the drug resistance by affecting the functions of transporters. It is importance to explore the potential mechanisms of AA in regulating the activity of the possible transporters. In addition, in vivo study should be included in the studying the regulatory effects of AA on the drug resistance by mediating the activity of MALAT1/β-catenin/MDR1 signaling.

## 5. Conclusion

Collectively, this study demonstrated the roles of MALAT1 and AA in the drug resistance of A549/DDP cells. Specifically, up regulated expression of MALAT1 was associated with β-catenin/MDR1 signaling-mediated drug resistance in A549/DDP cells. Knockdown of MALAT1 expression could ameliorate the drug resistance and increase the apoptosis of A549/DDP cells. Its possible underlying mechanism might be that MALAT1 up regulated the expression of MDR1 by sponging miR-1297, which targeted to degradation of p300. Overexpression of p300 could effectively compromise the knockdown of MALAT1 expression in the drug resistance of A549/DDP cells. AA enhanced DDP sensitivity in A549/DDP cells through decreasing MALAT1 level.

## Data Availability

Data supporting the research results can be accessed from the paper.
